The article "TLR4 Modulates Senescence and Paracrine Action in Placental Mesenchymal Stem Cells via Inhibiting Hedgehog Signaling Pathway in Preeclampsia" was retracted in 2025. Reasons: duplicated images; overlap with earlier publications; unreliable results or conclusions.

# TLR4 Modulates Senescence and Paracrine Action in Placental Mesenchymal Stem Cells via Inhibiting Hedgehog Signaling Pathway in Preeclampsia

**DOI:** 10.1155/2022/7202837

**Published:** 2022-06-14

**Authors:** Yanqi Zhong, Yang Zhang, Weifang Liu, Yin Zhao, Li Zou, Xiaoxia Liu

**Affiliations:** Department of Obstetrics and Gynecology, Union Hospital, Tongji Medical College, Huazhong University of Science and Technology, Wuhan, China

## Abstract

Preeclampsia (PE) is a heterogeneous disease closely associated with the accelerated senescence of the placentas. Placental mesenchymal stem cells (PMSCs) modulate placental development, which is abnormally senescent in PE together with abnormal paracrine. Both pivotal in the placenta development, Toll-like receptor 4 (TLR4) and Hedgehog (HH) pathway are also tightly involved in regulating cellular senescence. This study was aimed at demonstrating that TLR4/HH pathway modulated senescence of placentas and PMSCs *in vitro* and *in vivo*. Preeclamptic and normal PMSCs were isolated. Smoothed agonist (SAG) and cyclopamine were used to activate and inhibit HH pathway, respectively. Lipopolysaccharide (LPS) was used to activate TLR4 *in vitro* and establish the classic PE-like rat model. qRT-PCR, Western blotting, and immunofluorescence were used to detect the expression of TLR4 and HH components (SHH, SMO, and Gli1). Cellular biological function such as proliferation, apoptosis, and migration was compared. Cell cycle analysis, *β*-galactosidase staining, and the protein expressions of p16 and p53 were detected to analyze the cellular senescence. The secretion levels of human matrix metalloproteinase 9 (MMP-9) and soluble fms-like tyrosine kinase-1 (sFlt-1) were measured in the conditioned medium. Cell migration, invasion, and tube formation were analyzed in HTR8/SVneo cells or human umbilical vein endothelial cells (HUVECs). Our study demonstrated that activation of TLR4 accelerated senescence of PMSCs via suppressing HH pathway both *in vitro* and *in vivo*, accompanied by the detrimental paracrine to impair the uterine spiral artery remodeling and placental angiogenesis. Meanwhile, induction of HH pathway could alleviate PE-like manifestations, improve pregnancy outcomes, and ameliorate multiorgan injuries, suggesting that strengthening the HH pathway may serve as a potential therapy in PE.

## 1. Introduction

The well-developed placentation is fundamental for reproductive pregnancy and development of the fetus [1]. The defective placentation is the pathogenetic basis of multiple gestational disorders such as preeclampsia (PE) [1]. PE, one of the leading causes of maternal and perinatal morbidity and mortality [2], is a new-onset hypertension typically after 20 weeks of gestation, accompanied by multisystem signs or symptoms, including proteinuria, elevated liver enzymes, renal insufficiency, thrombocytopenia, and even maternal and fetal death [3]. Placental mesenchymal stem cells (PMSCs), a group of fibroblast-like cells with multipotential differentiation and self-renewal ability [4], are tightly involved in placentation via improving the uterine spiral artery remolding, augmenting the placental angiogenesis, and regulating the uteroplacental immune status [5–7]. On the contrary, preeclamptic PMSCs are dysfunctional with detrimental paracrine, thus playing a key role in the development and severity of PE [8–11]. Nonetheless, PMSCs are still a rather poorly understood cell type in the physiological functions of the placenta as well as the pathogenesis of PE.

Cellular senescence, a highly stable state of cell cycle arrest [12], is characterized by the induction of cyclin-dependent kinase inhibitors p16, tumor suppressor p53, and senescence-associated *β*-galactosidase (SA-*β*-gal) [13]. Moreover, senescent cells are characterized by abnormal paracrine secreting mixture of cytokines, chemokines, and matrix metalloproteins to influence the neighboring cells and microenvironment [14]. Although there exists the physiological senescence in the placenta as pregnancy advances to term [15], the preeclamptic placentas showed accelerated senescence [16–18]. Thereinto, preeclamptic PMSCs showed abnormal proliferation [19], arrested cell cycle [8], overexpressed p16, overactivated SA-*β*-gal, and abnormal secretory phenotype [11]. Furthermore, due to the detrimental paracrine actions, senescent PMSCs in PE have detrimental effects on trophoblasts and endothelial cells [11, 19], thus exacerbating the placental dysfunction. Nevertheless, the regulatory mechanisms of the cellular senescence in preeclamptic PMSCs remain to be elucidated.

Toll-like receptor 4 (TLR4) is the classic and pivotal receptor to trigger inflammatory and immune response [20]. Extensive research has reported that TLR4 is excessively activated and overexpressed in preeclamptic placentas [21] and tightly involved in the placental dysfunction [22]. However, studies have continuously proposed new association between TLR4 and other pathophysiological phenomenon in recent years, such as autophagy, metabolism reprogramming, and senescence [23, 24]. It has been demonstrated that the overexpression of TLR4 leads to cellular senescence in osteocyte and dental pulp stem cells [25–27]. Intriguingly, TLR4-activated bone marrow mesenchymal stem cells (BMMSCs) exhibit a similar secretory phenotype with the senescent PMSCs from preeclamptic placentas, such as interleukin(IL)-8 and soluble fms-like tyrosine kinase-1 (sFlt-1) [11, 28]. Nevertheless, whether the overactivated TLR4 in the PE placentas modulates cellular senescence in PMSCs remains to be clarified.

Hedgehog (HH) signaling pathway, an evolutionarily conserved pathway [29], involves three protein ligands including sonic Hedgehog (SHH), Indian Hedgehog (IHH), and desert Hedgehog (DHH) [30]. Once the ligands bind to the transmembrane receptor patched to inhibit the repression of Smoothened (Smo), Smo promotes Gli transcription factors (Gli1, Gli2, and Gli3) to translocate into the nucleus and regulate the transcription of the downstream targeting genes [31]. HH signaling pathway is pivotal in the development of the placenta [32] via regulating the trophoblastic invasion [33] and placental angiogenesis [34]. Besides, HH pathway was impaired in the placenta of PE [35]. Reportedly, HH pathway is tightly involved in regulating cellular senescence [36], especially the senescence of mesenchymal stem cells (MSCs) derived from various tissue [37, 38], while little was known about the role of HH pathway in PMSCs. Furthermore, the excessive activation of TLR4 contributes to the suppression of HH pathway in various cells with defective biological functions [39, 40]. Hence, it remains to be elucidated whether TLR4 regulates the senescence of PMSCs through HH pathway.

Lipopolysaccharide (LPS), a classic TLR4 agonist, has long been applied to induce *in vitro* and *in vivo* PE models for years [41–44]. In this study, we demonstrated that TLR4 activation regulates senescence of PMSCs via suppressing HH pathway *in vitro* and *in vivo*, leading to the dysfunction of trophoblasts and defective angiogenesis. Furthermore, the induction of HH pathway in LPS-induced PE rats ameliorated the PE-like manifestations and alleviated the placental senescence as well as PMSC senescence *in vivo*. Our study may provide new perspective for understanding the TLR4 in PE etiopathogenesis via modulating senescence in PMSCs. Furthermore, we indicated that the induction of HH pathway may be a novel and putative clinical management of PE.

## 2. Materials and Methods

### 2.1. Cell Isolation and Culture

PMSCs were isolated from placental tissue of normal pregnancies (*n* = 35) and preeclamptic pregnancies (*n* = 35) obtained from cesarean section. All of the study participants were from the Department of Obstetrics and Gynecology, Union Hospital, Wuhan, China and signed the informed consent. Ethical approval was obtained from the hospital's Ethics Committee (Ethics Code: S042). The clinical characteristics of the subjects were listed in Table 1. PE was diagnosed as the definition of American College of Obstetricians and Gynecologists [45], a new onset hypertension (systolic blood pressure sustained at ≥140 mmHg or diastolic blood pressure sustained at ≥90 mmHg, or both) with proteinuria, or end organ dysfunction after 20 weeks' gestation, or both [2]. The separation method was consistent with previous reports [5, 6]. Briefly, the placental tissue was washed twice with phosphate-buffered saline (PBS, Hyclone), the decidua and amniotic membrane were dissected apart carefully [46, 47], and the tissue was divided into 1 mm^3^ pieces. Then, the cut tissue was digested with 0.1 mg/mL collagenase type II (Sigma, USA) at 37°C for 1 h. The mixture was filtered through a 100 *μ*m cell strainer (Biosharp, China), and the filtrate was centrifuged at 2000 rpm for 25 mins to separate the PMSCs from the collagenase. The sediment was resuspended in DMEM F12 (Gibco, USA) containing 10% fetal bovine serum (FBS, Gibco). Then, the PMSCs were plated in 25 cm^2^ culture flasks and incubated at 37°C , 5% CO_2_ for three days. The medium was replaced every three days. To activate HH pathway, PMSCs were treated with 100 nM SAG [48] for 24 h as previously reported. To inhibit HH pathway, PMSCs were treated with 20 *μ*M cyclopamine [49] for 24 h as previously reported. For the TLR4-activated group, we added 200 ng/mL LPS (Sigma, USA) to culture the PMSCs for 24 h [21] as previously reported.

Human umbilical vein endothelial cells (HUVECs) were isolated from human umbilical cords collected from healthy donors via cesarean section as we reported previously [50]. The umbilical veins were washed with PBS and then digested with collagenase type I (Sigma, USA) for 15 min at 37°C. Then, HUVECs were collected by washing umbilical veins with complete endothelial cell medium (ECM) containing 10% FBS to stop digestion and centrifuged at 1000 rpm for 5 min. The sediment was resuspended in culture medium containing ECM and 10% FBS then incubated at 37°C, 5% CO_2_.

The immortalized human extravillous trophoblast (EVT) cell line HTR-8/SVneo was a kind gift from Dr. Charles Graham (Queen's University, Canada). Cells were cultured in 1640 (Gibco, USA) containing 10% FBS at 37°C containing 5% CO_2_.

### 2.2. Identification of PMSCs

The specific surface marker expression of PMSCs was evaluated by flow cytometry. PMSCs were digested with 0.25% trypsin-EDTA (Gibco, USA) and washed with PBS. PMSCs were incubated with PBS or fluorescein-labeled antibodies for 30 min. The tested antibodies included CD90, CD 105, CD73, CD44, CD34, CD31, and CD45 (Biolegend, USA) as previously reported [6, 51, 52]. Isotype-identical antibodies were used as controls. PMSCs were obtained in a fluorescence activated-cell sorter (Beckman, USA). Flow cytometric data were analyzed with FlowJo.v10.8.1 software. All experiments were performed at least three times.

### 2.3. Osteogenic, Adipogenic, and Chondrogenic Differentiation of PMSCs

For osteogenic, adipogenic, and chondrogenic differentiation, PMSCs were cultured in 6-well plates in differentiation medium (CYAGEN Biosciences, USA). The osteogenic differentiation medium contains basal medium supplemented with 10% FBS, 400 *μ*L ascorbate, 1% *β*-glycerophosphate, 20 *μ*L dexamethasone, 1% penicillin-streptomycin, and 1% glutamine. The PMSCs were stained with Alizarin Red (CYAGEN Biosciences, USA) and pictured with an optical microscope (Olympus, JAPAN). The adipogenic differentiation medium contains basal medium supplemented with 10% FBS, 400 *μ*L insulin, 200 *μ*L IBMX, 200 *μ*L dexamethasone, 1% L-glutamine, and 200 *μ*L rosiglitazone. After 21 days of culture, the PMSCs were fixed with 4% paraformaldehyde for 30 mins, then stained with Oil Red (CYAGEN Biosciences, USA), and pictured with an optical microscope. For chondrogenic differentiation, 4 × 10^5^ PMSCs were collected in a 15 mL centrifuge tube and were cultured in the chondrogenic differentiation medium (CYAGEN Biosciences, USA) as the instructions stated. After 21 days of culture, the cluster of PMSCs was fixed with 4% paraformaldehyde, embedded with paraffin, sliced into pieces, then stained with alcian blue (CYAGEN Biosciences, USA) staining, and pictured with an optical microscope. All experiments were performed at least three times.

### 2.4. Cell Proliferation Assay

Cell counting-8 (CCK-8) assay (C0038, Beyotime, China) was performed to measure the cell proliferation. Different groups of PMSCs were seeded on 96-well plates at a density of 8 × 10^3^/100 *μ*L cells per well. After 24 h/48 h/72 h, the 10 *μ*L CCK-8 solution was added to each well and the cells were incubated at 37°C. A multimode reader (Infinite F50; Tecan) measured the absorbance at 450 nm. All experiments were performed at least three times.

### 2.5. Apoptosis Analysis

Cell apoptosis was assessed using an Annexin V-FITC Apoptosis Detection Kit (BD Biosciences Pharmingen, San Diego, CA). Cells and supernatants were harvested, centrifuged, and washed with PBS. Then, the cells were resuspended with 100 *μ*L PBS and stained with 5 *μ*L annexin V and 5 *μ*L PI. The cells were incubated in the dark for 15 min and detected by a flow cytometry. Flow cytometric data were analyzed with FlowJo.v10.8.1 software. All experiments were performed at least three times.

### 2.6. Cell Cycle Analysis

The cell cycle assay was performed using a Cell Cycle Analysis Kit (C1052; Beyotime). The cells were harvested, washed with PBS, and fixed with 70% precooled ethanol at 4°C overnight. After being washed with PBS, the cells were stained with a mixture of propidium iodide, RNase A, and staining buffer for 30 mins in the dark. The cell cycle was detected by flow cytometry, and an analysis was performed by ModFitLT.v5 software. All experiments were performed at least three times.

### 2.7. Senescence-Associated *β*-galactosidase (SA-*β*-gal) Staining

The same passage of PMSCs was seeded in a 6-well plate, and *β*-galactosidase activity was tested by a Senescence *β*-galactosidase Staining Kit (C0602; Beyotime, China). Different groups of PMSCs were washed with PBS and fixed with fixative solution at room temperature for 15 min. Then, PMSCs were stained with mixture of staining solution according to manufacturer's instructions. After incubation at 37°C without CO_2_, PMSCs were washed with PBS and pictured under a microscope. Five fields were chosen randomly, and positive cells were counted. All experiments were performed three times.

### 2.8. Real-Time Quantitative PCR

Total RNA was extracted from the cells using TRIzol Reagent (Vazyme Biotech, Nanjing, China); then, RNA was used to construct cDNA using the HiScript III 1st Strand cDNA Synthesis Kit (Vazyme Biotech, Nanjing, China). Quantitative real-time PCR was performed using a StepOnePlus Real-Time PCR system (Applied Biosystems, CA, USA). The PCR cycling conditions were as follow: 95°C for 10 s, 60°C for 30 s, and 72°C for 30 s. *β*-Actin was used as an internal control to quantify mRNA expression. The primers are shown as follows:

*β*-Actin: F 5′-CATGTACGTTGCTATCCAGGC -3′; R 5′-CTCCTTAATGTCACGCACGAT -3′.

TLR4: F 5′-AGTTGATCTACCAAGCCTTGAGT-3′; R 5′-GCTGGTTGTCCCAAAATCACTTT-3′.

SHH: F 5′-GGACAAGTTGAACGCTTTGG-3′; R 5′-GCCCTCGTAGTGCAGAGACTC-3′.

SMO: F 5′-CAACCTGTTTGCCATGTTTG-3′; R 5′-TTTGGCTCATCGTCACTCTG-3′.

Gli1: F 5′-GGCAGCACTGAAGACCTCTC-3′; R 5′-ATTGGCCGGAGTTGATGTAG-3′.

All experiments were performed three times.

### 2.9. Western Blotting

Total proteins were extracted from cells with lysis buffer and were incubated for 15 min at 95°C. Then, proteins were subjected by 10% SDS-PAGE and then transferred to PVDF (polyvinylidene fluoride) membranes (0.45 *μ*m pore size; Millipore, MA, USA). The membranes were blocked with quick blocking buffer (P0252; Beyotime, China) for 10 min and then incubated with the anti-TLR4 (1 : 1,000; sc-293072; Santa Cruz), anti-SHH (1 : 1,000; 20697-1-AP; Proteintech), anti-SMO (1 : 2,000; ab266423; Abcam), anti-Gli1 (1 : 1,000; A14675; ABclonal), anti-p16 (1 : 1,000; A11651; ABclonal), anti-p53 (1 : 1,000; A19585; ABclonal), anti-MMP9 (1 : 1,000; 10375-2-AP; Proteintech), or anti-*β*- actin (1 : 4,000; 20536-1-AP; Proteintech) overnight at 4°C. The membranes were washed with TBST three times and then incubated with a secondary anti-rabbit antibody (1 : 4,000; GB23303; Servicebio) or anti-mouse antibody (1 : 4,000; GB23301; Servicebio) for 1 h. Finally, the membranes were visualized in chemiluminescence method (WVKLS0500; Millipore). All experiments were performed three times.

### 2.10. Conditioned Medium Preparation

After PMSCs were grown in DMEM F12 with 10% FBS until 80% confluent, the culture medium of PMSCs in different groups was removed. Cell layers were washed with PBS twice and subsequently incubated with serum-free DMEM F12 for 24 h in 37°C, 5% CO_2_. Then, the conditioned medium was collected and centrifuged at 2000 rpm for 10 min, filtered through a 0.22 *μ*m filter, and stored at −80°C for following experiments.

### 2.11. Enzyme-Linked Immunosorbent Assay (ELISA)

Conditioned media collected from different groups of PMSCs were prepared as mentioned. Human matrix metalloproteinase 9 (MMP-9), human soluble vascular permeability factor receptor 1/soluble fms-like tyrosine kinase-1 (sVEGFR1/sFlt1), rat matrix metalloproteinase 9 (MMP-9), and rat soluble vascular permeability factor receptor 1/soluble fms-like tyrosine kinase-1 (sVEGFR1/sFlt1) were measured in cell culture fluids using ELISA kits (Bioswamp, China), and the absorbance was quantified with a microplate reader (PerkinElmer chemagen, Germany) at 450 nm. The protein levels were calculated according to the standard curve. All experiments were performed three times.

### 2.12. Cell Migration Assay

Transwell units (24-well plates, 8 *μ*m pores; Corning Costar, NY, USA) were used to investigate the cell migration capacities. For PMSCs, different groups of PMSCs were resuspended in 200 *μ*L of serum-free medium and placed in the upper chamber, and 500 *μ*L complete medium was added to the lower chamber. The Transwell units were incubated in 37°C, 5% CO_2_ for 24 h. The units were stained with crystal violet (Servicebio, China) for 30 min; then, the cells were removed from the upper-membrane surface. Six fields were chosen randomly, and the number of the underside of the membrane was counted under a microscope.

Collected conditioned medium of different groups of PMSCs was added with 10% FBS additionally and then was used to pretreat HTR-8/SVneos and HUVECs for 24 h. The following migration steps were consistent with those mentioned before. All experiments were performed three times.

### 2.13. Cell Invasion Assay

Collected conditioned medium of different groups of PMSCs was added with 10% FBS additionally and then was used to pretreat HTR-8/SVneos for 24 h. Transwell units were coated with Matrigel (356234; BD Biosciences, USA) to investigate the cell invasion capacities. 100 *μ*L Matrigel was added to the upper chamber before the experiments and incubated at 37°C for 30 min, and then, the cells were suspended in serum-free medium, added 200 *μ*L to the upper chamber at a density of 2 × 10^5^/mL. The following steps were consistent with the cell migration assay. All experiments were performed three times.

### 2.14. Tube Formation Assay

Collected conditioned medium of different groups of PMSCs was added with 10% FBS additionally and then was used to pretreat HUVECs for 24 h. The 48-well plate was coated with 200 *μ*L/well Matrigel in advance. HUVECs (6 × 10^4^ cells/well) were resuspended in 200 *μ*L of complete medium and seeded in the 48-well plate with presolidified Matrigel. Tube-like structures were imaged with a microscope (Olympus; Japan), and the total length and branch points were analyzed using ImageJ software (NIH, Bethesda, MD, USA). All experiments were performed three times.

### 2.15. Immunofluorescence

The collected placental tissues were washed three times in PBS; then, tissues were embedded in paraffin and sliced into 5 *μ*m sections. After deparaffinization and antigen retrieval, sections were rehydrated in PBS for 15 minutes and then treated with PBS containing 0.1% of Triton X-100 and 1% of SDS for 4 minutes. Sections were washed in PBS for 5 minutes and blocked in 1% of BSA for 15 minutes. Sections were then incubated overnight in a humid chamber at 4°C with anti-TLR4 (1 : 100, 19811-1-AP, Proteintech), anti-SHH (1 : 100, 20697-1-AP, Proteintech), anti-SMO (1 : 200, ab266423, Abcam), anti-Gli1 (1 : 100, A14675, Abclonal), and anti-CD90 (1 : 200, ab181469, Abcam). Sections were washed in PBS three times for 5 min. Appropriate secondary antibodies were then applied for 1 h in the dark. Nuclei were stained with DAPI. PMSCs were labeled with anti-CD90 [53]. The sections were placed on the glass slides and were imaged by confocal microscopy (Nikon AIR SI Confocal; Nikon).

Different groups of PMSCs were seeded on coverslips and were fixed by 4% paraformaldehyde for 30 min. After blocking with 1% bovine serum albumin, PMSCs were incubated with anti-SMO (1 : 200; ab266423; Abcam) overnight. Then, PMSCs were incubated with secondary antibody, following with DAPI. Images were captured with a microscope and were analyzed by ImageJ.

All experiments were performed three times.

### 2.16. Animal and Experimental Design

The animal study was approved by the Institutional Ethics Review Board of Union Hospital, Tongji Medical College, Huazhong University of Science and Technology (Ethics Code: S2487). Sprague-Dawley (SD) rats were purchased form the Animal Center of Tongji Medical College. Female rats were raised in a light and humidity room (12 : 12 h) with abundant food and water, and they mated with male SD rats at 2 : 1 ratio. The presence of vaginal spermatozoa was used to confirm successful pregnancy and was designated as Gestational Day (GD) 0. Pregnant SD rats were divided into three groups: (1) the control group of SD rats (*n* = 7) was injected with saline at GD 13; (2) SD rats (*n* = 7) were injected with 20 *μ*g/kg LPS/body weight abdominally to create the PE-like model [54] at GD 13 until GD 18 as previously reported; and (3) SD rats (*n* = 7) were injected with the same dosage of LPS and further treated with 5 mM/kg SAG [55, 56] after 2 h as previously reported.

### 2.17. Detection of Blood Pressure, Urinary Protein, and Creatinine and Evaluation of Offspring Development

The systolic blood pressure (SBP) was assessed at GD 13 (before interference) and GD 19. The urine of rats was collected individually in metabolic cages without any food bur with free access to water, urinary protein was measured with a BCA protein assay kit (AS1086, Aspen, China), and creatinine was measured with the creatinine kit (C011-2-1, Jiancheng Biology, China). After sacrificing the rats, the length and weight of fetus and placentas were compared.

### 2.18. Tissue Collection and (Hematoxylin-Eosin) HE Staining

The rats were sacrificed using pentobarbital sodium anesthesia at GD 20. The placentas, livers, and kidneys were collected, washed, and fixed in 4% paraformaldehyde. Tissues were dehydrated through increasing alcohol concentration and embedded with paraffin. The 5 *μ*m paraffin sections of rats' placenta, liver, and kidney were cut and were stained with HE using standard protocols. All experiments were performed three times.

### 2.19. SA-*β*-gal Staining of Placentas

The placentas of rats were collected, washed by PBS, and stored in -80°C. The frozen slices of rats' placentas were stained with SA-*β*-gal kit (C0602; Beyotime, China) according to the manufacture's instruction.

### 2.20. Extraction and Identification of PMSCs in Rats

As previous researches have reported [57], the placentas of rats were collected and cut into small pieces. The remaining placental tissues were seeded into 25 cm^2^ culture flasks, and after 3 days, nonadherent cells were removed and the cultural media containing DMEM F12 and 10% FBS was replaced. The surface markers of PMSCs in rats were analyzed by flow cytometry. The tested antibodies included CD45 and CD90. The osteogenic, adipogenic, and chondrogenic differentiations were induced by osteogenic, adipogenic, and chondrogenic differentiation media (CYAGEN Biosciences, USA) as mentioned above.

### 2.21. Statistical Analysis

All data are presented as the mean ± SD, and statistical analyses were performed using GraphPad Prism 8.3.0 software (GraphPad Software). Unpaired Student's test was used to determine the significance of differences between the two groups. One-way ANOVA was used for multiple comparisons. *P* < 0.05 was considered significant. All experiments were performed at least three times.

## 3. Results

### 3.1. PMSCs Derived from Patients with PE Showed Accelerated Senescence along with Abnormal Paracrine

PMSCs adhered to cell culture plates after 3 days of culture, and the third passage of PMSCs showed fibroblastic morphology (Figure S1(a)). The expression of surface markers CD44, CD73, CD90, and CD105 was positive, while the expression of surface markers CD31, CD34, and CD45 was negative (Figure S1(b)), which was consistent with previous reports [6, 51, 52]. PMSCs also successfully formed calcified bone nodules, lipid droplets, and cartilage in the osteogenic, adipogenic, and chondrogenic differentiation assays (Figure S1(c)). Furthermore, we compared some biological functions between the normal PMSCs and preeclamptic PMSCs. Preeclamptic PMSCs showed poorer proliferation (*P* < 0.05; Figure 1(a)) but were not involved in apoptosis (Figure 1(b)) compared with the normal PMSCs. Preeclamptic PMSCs showed the increased percentage of cells in the G1/G0 phase (*P* < 0.001; Figure 1(c)) and the decreased percentage of cells in the S phase (*P* < 0.001; Figure 1(c)). The expressions of p16 (*P* < 0.01; Figure 1(d)) and p53 (*P* < 0.001; Figure 1(d)) were increased in the preeclamptic PMSCs. Moreover, preeclamptic PMSCs showed higher percentage of SA-*β*-gal positive cells (*P* < 0.01; Figure 1(e)). We further found that preeclamptic PMSCs showed weakened migration (*P* < 0.0001; Figure 1(f)) along with decreased expression of MMP9 protein (*P* < 0.01; Figure 1(g)). Conditioned media collected from preeclamptic PMSCs showed a lower level of MMP9 (*P* < 0.05; Figure 1(h)). Treated with conditioned media from preeclamptic PMSCs, HTR-8/SVneo cells exhibited deficient migration (*P* < 0.01; Figure 1(i)) and invasion (*P* < 0.01; Figure 1(j)) and a decreased protein expression of MMP9 (*P* < 0.01; Figure S2(a)). The impaired migration (*P* < 0.01; Figure 1(k)) along with decreased expression of MMP9 (*P* < 0.01; Figure S2(b)) was found in HUVECs when treated with conditioned media collected from the preeclamptic PMSCs. Besides, preeclamptic PMSCs secreted a higher level of sFlt-1 (*P* < 0.0001; Figure 1(l)). We further found that the total length of treated HUVECs was diminished (*P* < 0.01; Figure 1(m)).

### 3.2. Expression of TLR4 and the Hedgehog Pathway in Placentas and PMSCs of Both Preeclamptic and Normal Pregnancy

Preeclamptic placentas overexpressed TLR4 at both mRNA (*P* < 0.05; Figure S3(a)) and protein (*P* < 0.05; Figure 2(a)) levels. Representative immunofluorescent images of TLR4 expression in normal placentas and preeclamptic placentas showed the same results (Figure 2(b)). PMSCs from PE pregnancy showed increased expressions of TLR4 at mRNA (*P* < 0.05; Figure S3(d)) and protein (*P* < 0.01; Figure 2(f)) levels. Preeclamptic placentas exhibited lower expressions of main components of HH pathway (SHH, SMO, and Gli1) at mRNA (*P* < 0.05; Figure S3(b)-S3(d)) and protein levels (Figure 2(a)). Representative immunofluorescent images of SHH, SMO, and Gli1 expression in normal placentas and preeclamptic placentas showed the same results (Figures 2(c)–2(e)). Preeclamptic PMSCs expressed lower levels of SHH, SMO, and Gli1 at mRNA (Figure S3(f)-S3(h)) and protein (Figure 2(f)) levels. Hence, TLR4 was overexpressed and HH signal pathway was suppressed in the preeclamptic placentas and PMSCs.

### 3.3. TLR4 Modulated Cellular Senescence via Suppressing Hedgehog Pathway in PMSCs

The results of Western blottings (Figure 3(a)) and immunofluorescence (Figure 3(b)) showed the effectiveness of SAG and cyclopamine on regulating HH pathway. After treating PMSCs with LPS, PMSCs expressed lower levels of SHH (*P* < 0.01; Figure 3(a)), SMO (*P* < 0.05; Figure 3(a)) ,and Gli1 (*P* < 0.05; Figure 3(a)). When treated LPS-induced PMSCs with SAG, the expression levels of SMO (*P* < 0.01; Figure 3(a)) and Gli1 (*P* < 0.05; Figure 3(a)) were improved. Representative immunofluorescence images and quantification of double-fluorescent staining with SMO (red) and DAPI (blue) showed the same results (Figure 3(b)).

The results of CCK-8 showed that the induction of HH pathway promoted the cell proliferation (*P* < 0.0001; Figure 3(c)), and the inhibition of HH pathway showed opposite effects (*P* < 0.0001; Figure 3(c)). LPS-treated PMSCs exhibited significantly impaired (*P* < 0.0001; Figure 3(c)) proliferation, while SAG could reverse the inhibitory effect (*P* < 0.001; Figure 3(c)). The flow cytometry analysis showed that induction of HH pathway alleviated apoptosis (*P* < 0.05; Figure 3(d)), while inhibition of the HH pathway did not involve in apoptosis. The apoptosis was not significantly changed in LPS-treated PMSCs.

The inhibition of the HH pathway increased the cell percentage of the G1/G0 phase (*P* < 0.01; Figure 3(e)) and decreased the cell percentage of the S phase (*P* < 0.05; Figure 3(e)). LPS-treated PMSCs displayed a remarkably higher percentage of cells in the G1/G0 phase (*P* < 0.001; Figures 3(e)) and a lower percentage of cells in the S phase (*P* < 0.01; Figure 3(e)), while SAG could reverse this effect.

Both inhibition of the HH pathway and induction by LPS showed augmented expression levels of p16 (Figure 3(f)) and p53 (Figure 3(f)) in PMSCs. However, treating LPS-stimulated PMSC with SAG expressed lower protein levels of p16 (*P* < 0.01; Figure 3(f)) and p53 (*P* < 0.05; Figure 3(f)). The detection of SA-*β*-gal showed the same trend (Figure 3(g)) as expressions of p16 and p53.

Induction of HH pathway could promote the migration (*P* < 0.05; Figure 3(h)) and increased the protein expression levels of MMP9 (*P* < 0.001; Figure 3(i)). Conversely, inhibition of HH pathway showed opposite effects (Figures 3(h) and 3(i)). LPS stimulation impaired the migration (*P* < 0.01; Figure 3(h)) and diminished the protein expression of MMP9 (*P* < 0.001; Figure 3(i)), while SAG could improve the effects.

### 3.4. TLR4/Hedgehog Pathway Mediated the Paracrine Action of PMSCs, Affecting the Functions of Trophoblasts and HUVECs

The conditioned media from different groups were collected to measure the secretion levels of MMP9 and treat HTR-8/SVneo cells. After activating HH pathway, the conditioned media collected from PMSCs showed a higher level of MMP9 (*P* < 0.0001; Figure 4(a)), promoted the of trophoblastic migration (*P* < 0.05; Figure 4(b)) and invasion (*P* < 0.0001; Figure 4(c)) along with the elevated expression of MMP9 (*P* < 0.01; Figure S2(c)), and promoted migration of HUVEC (*P* < 0.001; Figure 4(d)) with increased level of MMP9 (*P* < 0.001; Figure S2(d)). Inhibition of HH pathway exhibited opposite effects. LPS-stimulated PMSCs secreted a lower level of MMP9 (*P* < 0.01; Figure 4(a)), the conditioned media of which suppressed the migration (*P* < 0.001; Figure 4(b)) and invasion (*P* < 0.0001; Figure 4(c)) of HTR-8/SVneo cells with diminished levels of MMP9 (*P* < 0.01; Figure S2(c)), impaired migration of HUVECs (*P* < 0.0001; Figure 4(d)) with decreased expression of MMP9 (*P* < 0.05; Figure S2(d)), while SAG reversed these inhibitory effects.

The secretion levels of sFlt-1 were measured, and the conditioned media were collected to treat HUVECs. The conditioned media of PMSCs with the suppressed HH pathway had a higher level of sFlt-1 (*P* < 0.001; Figure 4(e)) and weakened the tube formation of HUVECs (Figure 4(f)). LPS-stimulated PMSCs showed the same trend as inhibition of HH pathway; however, these effects were reversed by SAG.

### 3.5. Activation of the Hedgehog Pathway Ameliorated PE Manifestations, Pregnancy Outcomes, and Organ Injuries in LPS-Induced PE-Like Rats

To investigate the potential role of the HH pathway in PE, we established a PE-like rat model induced by LPS (LPS group) and injected SAG into the rats of the LPS group (SAG group). The schematic diagram of the animal experimental design was showed in Figure 5(a). The maternal weight gain of pregnant rats was not significance (Figure 5(b)) among the groups. In the rats treated with LPS, we found an increased SBP (*P* < 0.05; Figure 5(d)), proteinuria (*P* < 0.001; Figure 5(f)), and creatinine (*P* < 0.001; Figure 5(h)) post injection (GD19) compared with the control group (saline), which were reduced via the SAG administration. Furthermore, the fetus of the rats (Figure 5(k)) treated with LPS showed lower fetal weight (*P* < 0.0001; Figure 5(i)) and reduced fetal length (*P* < 0.0001; Figure 5(j)) compared with the saline group, while SAG revered the maldevelopment of the fetus. The placentas (Figure 5(n)) from the LPS-induced rats showed shorter placental diameters (*P* < 0.0001; Figure 5(l)) and lower placental weights (*P* < 0.05; Figure 5(m)). After administration of SAG, the placentas' size was improved (*P* < 0.05; Figures 5(l) and 5(m)). The rate of premature birth and still birth is shown in Table 2. HE staining of placentas in the LPS group showed villous cellulose-like necrosis, narrowing of vascular lumen (Figure 5(o)). HE staining of liver tissues showed LPS induced hepatocyte steatosis, ballooning degeneration of the hepatocytes (Figure 5(p)). The renal tissues showed LPS contributed to the collapse of tubular epithelial cells (Figure 5(q)). These histological changes were not observed in the control group and the SAG group.

### 3.6. Activation of the Hedgehog Pathway Regulated the Senescence of Placentas and PMSCs in LPS-Induced PE-Like Rats

We collected placentas from the pregnant rats. The expression of TLR4 was higher (*P* < 0.001; Figure 6(a)) in the placentas of the LPS group compared with the control group, and the expression of TLR4 was not significant in the placentas of the LPS group and SAG group. The expressions of SMO (*P* < 0.01; Figure 6(a)) and Gli1 (*P* < 0.001; Figure 6(a)) were downregulated in the placentas of the LPS group, while the expression of SMO (*P* < 0.001; Figure 6(a)) and Gli1 (*P* < 0.0001; Figure 6(a)) was upregulated in the placentas of the SAG group. To assess the senescence in placentas, we found the protein expressions of p16 (*P* < 0.01; Figure 6(b)) and p53 (*P* < 0.01; Figure 6(b)), and the activity SA-*β*-gal (Figure 6(c)) were elevated in the placentas of the LPS group, while SAG administration alleviated the placental senescence.

We extracted the PMSCs of rats (Figure 6(d)), identified the osteogenic, adipogenic, and chondrogenic differentiation ability of PMSCs (Figure 6(e)), and analyzed the negative surface marker (CD45) and the positive surface marker (CD90) of PMSCs (Figure 6(f)) as previously reported [58]. The expressions of TLR4 and the HH pathway components (SMO and Gli1) in PMSCs from LPS-induced rats were consistent with the placentas (Figure 6(g)). Moreover, the expressions of p16 (*P* < 0.01; Figure 6(h)) and p53 (*P* < 0.05; Figure 6(h)) were higher in the PMSCs from LPS-induced rats, and administration of SAG could ameliorate the levels of cellular senescence in rat PMSCs. The detection of SA-*β*-gal showed the same trend as the expressions of p16 and p53 (Figure 6(i)). Senescent rat PMSCs also showed abnormal paracrine action. The conditioned media collected from the PMSCs of the LPS group showed a lower level of MMP9 (*P* < 0.001; Figure 6(j)) and a higher level of sFlt-1 (*P* < 0.05; Figure 6(k)). The PMSCs of the SAG group secreted a higher level of MMP9 (*P* < 0.01; Figure 6(j)) and a lower level of sFlt-1 (*P* < 0.05; Figure 6(k)) compared with the LPS group.

## 4. Discussion

The precise pathogenesis of PE remains vague and complicated while the prevailing hypothesis centers on defective early placental development [59]. Dysfunctions of PMSCs are linked with the development of PE [60]. Based on previous study, preeclamptic PMSCs showed accelerated senescence accompanied by aberrant secretory phenotype, thus having detrimental effects on adjacent cells in the placenta [11]. In this study, we further verified that preeclamptic PMSCs were more senescent and exhibited detrimental paracrine, thus impairing trophoblastic invasion and endothelial angiogenesis. Moreover, we found that the expression of TLR4 was significantly increased while the expressions of the HH pathway (SHH, SMO, and Gli1) were significantly decreased both in the preeclamptic placentas and preeclamptic PMSCs. Mechanically, we demonstrated that TLR4/HH pathway modulated senescence of PMSCs, contributing to abnormal secretory phenotype *in vivo* and *in vitro* to affect spiral artery remodeling and placental angiogenesis.

Although physiological senescence of placentas is inevitable in normal pregnancy [15], preeclamptic placentas showed abnormally accelerated senescence. [61]. Biron et al. found that preeclamptic trophoblasts showed abnormal senescence with shorter telomere lengths [62]. Cecati et al. demonstrated that the reduction of Klotho expression accelerated senescence of the preeclamptic placenta [63]. In our study, we found that preeclamptic PMSCs showed accelerated senescence with dysfunction, which is consistent with the previous research [11]. As cellular senescence is characterized by abnormal paracrine [13], we further verified that preeclamptic PMSCs in our study had detrimental paracrine action on trophoblasts and ECs. Thereinto, we focused on MMP9 and sFlt-1 which correlate strongly with the pathogenesis of PE. MMP9, degrading extracellular matrix to enhance cell migration and invasion, is particularly prominent for spiral artery remodeling [64]. Our results showed that preeclamptic PMSCs secreted lower levels of MMP9, which weakened the trophoblastic migration and invasion. Similarly, sFlt-1, one of the antiangiogenic factors, causes endothelial dysfunction in PE [65, 66]. In this study, we found that the conditioned media of preeclamptic PMSCs contained higher levels of sFlt-1, which impaired the migration and angiogenesis of ECs. Hence, compared with normal PMSCs, we found that preeclamptic PMSCs exhibited accelerated senescence, further affecting the crosstalk with adjacent cells through abnormal paracrine. Yet the exact regulatory mechanism of senescence of preeclamptic PMSCs remains vague.

It is widely acknowledged that TLR4 overactivation at the uteroplacental interface causes placental dysfunction in PE [67] via shallowing the trophoblastic invasion [21] and suppressing the ability of angiogenesis in ECs [68]. Nevertheless, the expression of TLR4 in preeclamptic PMSCs remains vague, while our data indicated that preeclamptic PMSCs were TLR4 activated. TLR4 activation also induced cellular senescence in various cells [25–27, 69]. Reportedly, TLR4-activated neurons showed increased expression of p53, elevated SA-*β*-Gal, and remarkable cell cycle arrest [26]. TLR4-activated alveolar bone osteocytes showed upregulated mRNA expression of p16, p21, and p53, overexpressed SASP factors, and severe DNA damage [25]. In our study, after treated with low-dose of LPS [21], TLR4-activated PMSCs were accelerated senescence with arrested cell cycle, overexpressed p16 and p53, and higher activity of SA-*β*-Gal. Moreover, with the activation of TLR4, the senescent PMSCs had detrimental effects on trophoblasts and ECs via abnormal paracrine. However, the underlying mechanism how TLR4 regulated senescence in PE PMSCs needs further investigation.

HH signaling pathway played a crucial role in mediating senescence [38]. Based on previous study, induction of the HH pathway can function as an antagonist of senescence [38] via promoting DNA repair and reducing oxidative stress [70]. Conversely, suppression of HH pathway leads to senescent hallmarks such as overexpressed p16, p53, and abnormal secretory phenotype [37]. Consistent with previous study [32], we found that the main components of HH pathway were downregulated in the preeclamptic placenta and preeclamptic PMSCs. We demonstrated that the suppression of HH pathway accelerated senescence of PMSCs. Reportedly, TLR4 activation can partly inhibit HH pathway both *in vivo* [71] and *in vitro* [39, 40]. Intraamniotic LPS exposure decreased the expression of HH pathway in the ovine fetus [71]. Treated with LPS, neurons [40] and brain-microvascular endothelial cells [39] both showed downregulation with HH pathway along with dysfunctions. Our study also indicated that the TLR4-mediated HH pathway accelerated senescence of PMSCs along with abnormal paracrine, contributing to deficient spiral artery remodeling and defective angiogenesis. Therefore, we demonstrated that the activation of TLR4 accelerated the senescence of PMSCs via suppressing HH pathway *in vitro*.

Furthermore, in order to verify that TLR4 modulated senescence of PMSCs via suppressing HH pathway *in vivo*, we established the PE-like rat model by injecting LPS and treated the LPS-induced rats with SAG. The rats of the SAG group showed alleviated PE-like manifestations, improved pregnancy outcomes, and ameliorated multiorgan injuries in our study. It was reported that targeting HH pathway improved the blood pressure, angiogenic imbalance, inflammation, and pregnancy outcome in reduced uterine perfusion pressure (RUPP) model of PE rats [72]. Hence, our study further indicated that the induction of HH pathway would be a potential clinical management in PE. Moreover, the placentas and PMSCs of PE model rats were accelerated senescent, while the senescence of placenta and PMSCs was reversed via HH activation. These findings suggested that TLR4/HH pathway modulated senescence of PMSCs *in vivo*, results of which were consistent with our *in-vitro* study.

In conclusion, our investigation demonstrated that TLR4 activation suppressed HH pathway in preeclamptic PMSCs, thus leading to accelerated senescence of PMSCs, along with the abnormal paracrine to impair the function of trophoblasts and angiogenesis at the uteroplacental interface of PE both *in vitro* and *in vivo*. Our findings may provide new insights into the pathogenesis of PE and indicated that the HH pathway may be a novel and potential clinical management of PE.

## 5. Conclusion

Our study demonstrated that activation of TLR4 accelerated senescence of PMSCs via suppressing HH pathway both *in vitro* and *in vivo*, accompanied by the detrimental paracrine to impair the uterine spiral artery remodeling and placental angiogenesis. However, induction of HH pathway could reverse those negative effects, suggesting that strengthening the HH pathway may serve as the potential therapies in PE through suppressing the senescence of placentas and PMSCs.

## Figures and Tables

**Figure 1:** The dysfunctions of preeclamptic PMSCs and their detrimental effects on trophoblasts and HUVECs. (a) The proliferation of normal PMSCs and preeclamptic PMSCs using CCK-8 assays. (b) The apoptotic rates of normal PMSCs and preeclamptic PMSCs using flow cytometry assays. (c) The cell cycle phases of normal PMSCs and preeclamptic PMSCs were determined using flow cytometry assays. (d) Western blot analysis and densitometric quantification of p16 and p53 protein expressions in the normal PMSCs and preeclamptic PMSCs. (e) SA-*β*-gal staining of PMSCs and the average ratio of SA-*β*-gal-positive cells in the normal PMSCs and preeclamptic PMSCs. (f) Representative Transwell photos of PMSCs as well as the relative PMSCs number of the Transwell quantified. (g) Western blot analysis and densitometric quantification of MMP9 protein expression in the normal PMSCs and preeclamptic PMSCs. (h) ELISA analysis of MMP9 concentrations of cell culture medium in the preeclamptic and normal PMSCs. (i) Representative Transwell photos and cell number of the migrated HTR-8/Svneo cells in different groups. (j) Representative Transwell photos and cell number of the invasive HTR-8/Svneo cells in different groups. (k) Representative Transwell photos and the cell number of the HUVEC migration in different groups. (l) ELISA analysis of sFlt-1 concentrations of cell culture medium in the preeclamptic and normal PMSCs. (m) Tube formation of HUVECs and the total length of the formative tube in different groups. Scale bar: 200 *μ*m. Data are presented as the mean ± SD. ^∗^*P* < 0.05, ^∗∗^*P* < 0.01, ^∗∗∗^*P* < 0.001, and ^∗∗∗∗^*P* < 0.0001 by Student's *t*-test. SD: Standard deviation.

**Figure 2:** The expressions of TLR4 and HH pathway components (SHH, SMO, and Gli1) in the placentas and PMSCs from the patients with PE. (a) Western blot analysis of TLR4, SHH, SMO, and Gli1 protein expression and quantitative analysis of TLR4, SHH, SMO, and Gli1 in the normal and preeclamptic placentas. Protein data were normalized to *β*-actin. (b)–(e) Double labeling the immunofluorescence analysis of TLR4 (b), SHH (c), SMO (d), and Gli1(e) protein expression and localization in the placentae from full-term normal pregnancies and preeclampsia patients. TLR4, SHH, SMO, and Gli1 (red). DAPI (blue). CD90 (green) for PMSCs localization. (f) Western blot analysis of TLR4, SHH, SMO, and Gli1 protein expression and quantitative analysis of TLR4, SHH, SMO, and Gli1 in the normal and preeclamptic PMSCs. Scale bar: 200 *μ*m. Data are presented as the mean ± SD. ^∗^*P* < 0.05, ^∗∗^*P* < 0.01, ^∗∗∗^*P* < 0.001, and ^∗∗∗∗^*P* < 0.0001 by Student's *t*-test. SD: Standard deviation.

**Figure 3:** LPS-induced TLR4 activation modulates functions of PMSCs via suppressing HH pathway. PMSCs were treated with SAG, cyclopamine, LPS and LPS+SAG separately. (a) Western blot analysis (a) of TLR4, SHH, SMO, and Gli1 protein expression and quantitative analysis of TLR4, SHH, SMO, and Gli1 in different groups of PMSCs. (b) Representative immunofluorescence images and quantification of double-fluorescent staining with SMO (red) and DAPI (blue). (c) CCK-8 assays were performed to determine the proliferation in different groups of PMSCs. (d) The apoptotic rates in different groups of PMSCs using flow cytometry assays. (e) The cell cycle phases of different groups of PMSCs were determined using flow cytometry assays. (f) Western blot analysis and densitometric quantification of p16 and p53 protein expressions in different groups of PMSCs. (g) SA-*β*-gal staining of PMSCs and the average ratio of SA-*β*-gal-positive cells in different groups of PMSCs. (h) Representative Transwell photos of PMSCs as well as the relative PMSC numbers of the Transwell quantified in different groups. (i) Western blot analysis and densitometric quantification of MMP9 protein expression in different groups of PMSCs. Scale bar: 200 *μ*m. Data are presented as the mean ± SD. ^∗^*P* < 0.05, ^∗∗^*P* < 0.01, ^∗∗∗^*P* < 0.001, and ^∗∗∗∗^*P* < 0.0001 by Student's *t*-test and one-way ANOVA. SD: Standard deviation.

**Figure 4:** Effects of the conditioned media of TLR4/HH pathway regulated PMSCs on HTR-8/Svneo cells and HUVECs. (a) ELISA analysis of MMP9 concentrations of cell culture medium in different groups of PMSCs. (b) Representative Transwell photos and cell number of the migrated HTR-8/Svneo cells in different groups. (c) Representative Transwell photos and cell number of the invasive HTR-8/Svneo cells in different groups. (d) Representative Transwell photos and the cell number of the HUVEC migration in different groups. (e) ELISA analysis of sFlt-1 concentrations of cell culture medium in the preeclamptic and normal PMSCs. (f) Tube formation of HUVECs and the total length of the formative tube in different groups. Scale bar: 200 *μ*m. Data are presented as the mean ± SD. ^∗^*P* < 0.05, ^∗∗^*P* < 0.01, ^∗∗∗^*P* < 0.001, and ^∗∗∗∗^*P* < 0.0001 by Student's *t*-test and one-way ANOVA. SD: Standard deviation.

**Figure 5:** Intervention effects of SAG on LPS-induced preeclamptic features. (a) Schematic diagram of the animal experimental design. (b) Effects of SAG and LPS on maternal body weight gain. *Δ*Maternal body weight: the increased body weight referring to GD0 as baseline. (c) and (d) SBP of GD13 (c) and GD19 (d) in different groups of rats. (e) and (f) Proteinuria of GD13 (e) and GD19 (f) in different groups of rats. (g) and (h) Creatinine of GD13 (g) and GD19 (h) in different groups of rats. (i)–(k) Fetal development in each group. Fetal weight (i) and fetal length (j) in different groups. (l)–(n) Placental size in each group. Placental diameters (l) and placental weight (m) in different groups. (o) HE staining of placenta tissues in different groups of rats. (p) HE staining of liver tissues in different groups of rats. (q) HE staining of kidney tissues in different groups of rats. Scale bar: 200 *μ*m. Data are presented as the mean ± SD. ^∗^*P* < 0.05, ^∗∗^*P* < 0.01, ^∗∗∗^*P* < 0.001, and ^∗∗∗∗^*P* < 0.0001 by Student's *t*-test. SD: Standard deviation.

**Figure 6:** SAG reversed the senescence degree of the placentas and PMSCs in the LPS-induced rats. (a) Western blot analysis of TLR4, SMO, and Gli1 protein expression and quantitative analysis of TLR4, SMO, and Gli1 in different groups of placentas. (b) Western blot analysis and densitometric quantification of p16 and p53 protein expressions in different groups of placentas. (c) SA-*β*-gal staining of the placentas of different groups of rats. (d) Morphology of rat PMSCs. Small fibroblast- like MSC colonies were detected by an inverted microscope. (e) Successfully differentiated PMSCs of rats were stained with Alizarin Red for osteogenic differentiation, Oil Red O for adipocytes, and alcian blue, in which red calcium nodules, orange lipid droplets, and blue cartilage could be observed. (f) PMSCs of rats expressed CD90 but not CD45. (g) Western blot analysis of TLR4, SMO, and Gli1 protein expression and quantitative analysis of TLR4, SMO, and Gli1 in different groups of PMSCs. (h) Western blot analysis and densitometric quantification of p16 and p53 protein expressions in different groups of placentas. (i) SA-*β*-gal staining of different groups of rat PMSCs and the average ratio of SA-*β*-Gal-positive cells in different groups of PMSCs. (j) ELISA analysis of MMP9 concentrations of cell culture medium in different groups of PMSCs. (k) ELISA analysis of sFlt-1 concentrations of cell culture medium in different groups of PMSCs. Scale bar: 200 *μ*m. Data are presented as the mean ± SD. ^∗^*P* < 0.05, ^∗∗^*P* < 0.01, ^∗∗∗^*P* < 0.001, and ^∗∗∗∗^*P* < 0.0001 by Student's *t*-test. SD: Standard deviation.

**Table 1:** Clinical characteristics of study population.

Parameters	Normal (*n* = 35)	Preeclampsia (*n* = 35)	*P* value preeclampsia vs. Normal
Maternal age (year)	32.0 ± 4.2	32.8 ± 0.7	*P* > 0.05
BMI in pregnancy (kg/m^2^)	26.9 ± 1.4	29.3 ± 4.6	*P* > 0.05
Gestational age (week)	38 ± 0.7	34 ± 2.9	*P* < 0.05
Systolic blood pressure at delivery (mmHg)	120 ± 6.0	155 ± 11.7	*P* < 0.05
Diastolic blood pressure at delivery (mmHg)	75 ± 6.9	103 ± 8.9	*P* < 0.05
Proteinuria (g/day)	0 (0/35)	100 (35/35)	*P* < 0.05
Body weight of infant (g)	3303 ± 460	2018 ± 879	*P* < 0.05

Data are presented as mean ± SD or percentage (number/total). *P* value <0.05 was considered as significant difference. BMI: Body mass index in pregnancy (kg/m^2^); proteinuria (quantity of 24 h urine protein excretion) higher or equal to 300 mg/24 h is proteinuria positive and lower than 300 mg/24 h is proteinuria negative.

**Table 2:** Pregnancy outcomes in different pregnant groups.

	Saline (*n* = 7)	LPS (*n* = 7)	LPS+SAG (*n* = 7)
Litter size	14.14 ± 1.35	12.57 ± 1.51	13.85 ± 1.07
Premature birth (%)	0 (0/99)	13.63 (12/88)^∗∗∗^	0 (0/97)^∗∗∗^
Stillbirth (%)	0 (0/99)	7.96 (7/88)^∗∗^	0 (0/97)^∗∗^
Fetal weight (g)	5.78 ± 0.36	3.62 ± 0.51^∗∗∗∗^	6.63 ± 0.77^∗∗∗∗^
Fetal length (cm)	4.31 ± 0.18	3.19 ± 0.44^∗∗∗∗^	4.58 ± 0.24^∗∗∗∗^
Placental weight (g)	0.50 ± 0.08	0.43 ± 0.05^∗^	0.47 ± 0.09
Placental diameters (cm)	1.70 ± 0.14	1.40 ± 0.09^∗∗∗∗^	1.55 ± 0.15^∗^

Data are presented as mean ± SD or percentage (number/total). ^∗^*P* < 0.05, ^∗∗^*P* < 0.01, ^∗∗∗^*P* < 0.001, and ^∗∗∗∗^*P* < 0.0001 (LPS versus saline; LPS+SAG versus LPS).

## Data Availability

The data are included in the article to support the findings of this study.

## Supplementary Materials

Supplementary 1
*Figure S1*. Morphology, differentiation, and surface markers of PMSCs. (a) PMSC morphology was detected by an inverted microscope. Three and fourteen days after isolation, small fibroblast-like MSC colonies were visible. Cell culture was enriched in a population of cells characterized by a fibroblast-like spike appearance at 100x magnification. (b) Successfully differentiated PMSCs were stained with Alizarin Red for osteogenic differentiation, Oil Red O for adipocytes, and alcian blue, in which red calcium nodules, orange lipid droplets, and blue cartilage could be observed. (c) PMSC surface markers. PMSCs expressed CD44, CD73, CD90, and CD105 but not CD31, CD34, and CD45. Scale bar: 200 *μ*m.

Supplementary 2
*Figure S2*. Protein expressions of MMP9 in HTR-8/Svneo cells and HUVECs treated with the conditioned media of different groups of PMSCs. (a) Western blot analysis as well as the densitometric quantification of MMP9 protein expression of HTR-8/Svneo cells treated with the conditioned media of preeclamptic PMSCs and normal PMSCs. (b) Western blot analysis as well as the densitometric quantification of MMP9 protein expression of HUVECs treated with the conditioned media of preeclamptic PMSCs and normal PMSCs. (c) Western blot analysis as well as the densitometric quantification of MMP9 protein expression of HTR-8/Svneo cells in different groups. (d) Western blot analysis as well as the densitometric quantification of MMP9 protein expression of HUVECs in different groups. Data are presented as the mean ± SD. ^∗^*P* < 0.05, ^∗∗^*P* < 0.01, ^∗∗∗^*P* < 0.001, and ^∗∗∗∗^*P* < 0.0001 by Student's *t*-test and one-way ANOVA. SD: Standard deviation.

Supplementary 3
*Figure S3*. The mRNA expressions of TLR4 and HH pathway components (SHH, SMO, and Gli1) in the placentas and PMSCs from patients with PE. (a) qRT-PCR analysis of TLR4 mRNA levels of the placentas with PE and normal pregnancy. (b-d) qRT-PCR analysis of SHH (b), SMO (c), and Gli1(d) mRNA levels of the placentas with PE and normal pregnancy. (e) qRT-PCR analysis of TLR4 mRNA levels of the PMSCs from the placentas with PE and normal pregnancy. (f-h) qRT-PCR analysis of SHH (f), SMO (g), and Gli1(h) mRNA levels of the PMSCs from the placentas with PE and normal pregnancy. Data are presented as the mean ± SD. ^∗^*P* < 0.05, ^∗∗^*P* < 0.01, ^∗∗∗^*P* < 0.001, and ^∗∗∗∗^*P* < 0.0001 by Student's *t*-test. SD: Standard deviation.
